The article "Grape Leaf Disease Classification Combined with U-Net++ Network and Threshold Segmentation" was retracted in 2023. Reasons: unreliable results or conclusions; concerns about the data; concerns about the peer review; concerns about the citations.

# Grape Leaf Disease Classification Combined with U-Net++ Network and Threshold Segmentation

**DOI:** 10.1155/2022/1042737

**Published:** 2022-10-07

**Authors:** Guowei Wang, Jiawei Wang, Jiaxin Wang, Yadong Sun

**Affiliations:** College of Information Technology, Jilin Agricultural University, Changchun 130118, China

## Abstract

Applying the method of semantic segmentation to the segmentation of grape leaves is an important method to solve how to segment grape leaves from complex backgrounds. This article uses U-net++ convolutional neural network to segment grape leaves from complex backgrounds using MIOU, PA, and mPA as evaluation metrics. After the leaves are segmented, the OTSU threshold segmentation + EXG algorithm is used to extract the diseased spots of grape leaves and healthy grape leaves by increasing the proportion of green vectors. Grape leaf disease was automatically graded by the ratio of the healthy green part of the grape to the total leaf area.

## 1. Introduction

China is the world's second-largest grape planting area and the world's largest grape production country. Grape leaf diseases such as grape black rot, grape brown spot, grape ring spot, and other leaf diseases seriously threaten the yield of grapes in my country and cause significant economic losses [1]. The traditional segmentation research on grape leaf diseases and even the segmentation research on disease images in the entire plant leaf field all have empirical judgments, which are time-consuming and labor-intensive. With the development of computer vision technology and the rapid application of deep learning in the computer field, it is possible to conduct rapid and effective research on grape leaf diseases, which is of great significance to the research on grape diseases [2, 3].

At present, the research on plant leaf diseases mainly focuses on the fields of disease feature extraction and disease segmentation. Image segmentation is the key difficulty in solving the above problems. When collecting grape leaves, the leaves will be affected by various noises such as light, background, and shadow. So how to accurately segment the grape leaves under such a complex background and study the diseases of the segmented grape leaves has become a practical problem to be solved [2–6].

This article will focus on grape leaves as the research object, deal with the top diseases of grape leaves, take the segmentation of leaves in complex environments as the operation content, and combine deep learning and threshold segmentation. First, deep learning is used, and the U-net++ convolutional neural network is selected to remove the complex environment of the picture and segment the grape leaves from the complex environment. The segmented grape leaves were segmented by the OTSU method, and the grape diseases were segmented from the leaves. The OTSU threshold segmentation first performs binarization processing on the image. After the binarization processing, the EXG algorithm is used to enhance the green vector part in the segmented grape leaves, and the green part of the image is segmented from the grape disease. This article provides a feasible method for the segmentation of plant leaves including grape leaves and plant leaf diseases in complex backgrounds.

## 2. Data Collection

The data used in this article come from the 2018 AI changer competition and the use of a Canon 500 camera to shoot the leaves at a vertical distance of about 30 cm. The camera is set to unify automatic focus, pay attention to turning off the flash function to avoid exposure that affects the white balance, ensure that the grape leaves are clear and complete, and store the images in .jpg format. The three types of grape leaf diseases were black rot, ring spot, and brown spot.

The image needs to be marked first, and the next operation can be performed after marking the image. The image labeling tool we chose is labelme, which accurately labels grape leaves.

The grape leaves are marked in the picture. The labeling process is shown in Figure 1. Polygons are created on the picture and the grape leaves of the entire label are marked. After the annotation is completed, a .json file will be generated for each image, and the data for training will be generated after processing the .json file.

## 3. Segmentation of Grape Leaves in Complex Environment

For a convolutional neural network, if it can identify different positions and directions of the same object, we call this convolutional network an invariant convolutional neural network. The methods of data enhancement mainly include flipping, rotating, scaling, shifting, and Gaussian noise reduction.

For segmentation of grape leaf disease, in this article, the deep learning method is adopted, and the U-net++ network structure is used to segment the grape leaves from the complex environment so that the study of grape disease spots is based on the output map of the U-net++ network structure model.

### 3.1. U-Net++ Network

Semantic segmentation is the key to solving the segmentation of grape leaves under complex background in this article. Grape leaves can be segmented from an environment with similar background and foreground colors and no obvious color difference and complex background [5, 7, 8]. In 2015, the fully convolutional network was developed, and image segmentation has made great progress. Then the development of U-net can get better results with very little data.

U-net++ was developed in 2018. U-net++ is essentially an encoder-decoder (encode-decode) network [7–9]. The long connections in the U-net network are removed and replaced by a series of short links. It is a comprehensive long connection. About the short connection scheme, it captures different features, superimposes and fuses their features, and has different degrees of sensitivity to different target models. In the actual semantic segmentation operation process, about the edge feature extraction of large objects and small objects, it is easy to be lost by the downsampling and upsampling of the deep network. At this time, you can need the help of the small feature of the perception field. The encoder of U-net++ in this article uses the ResNet18 residual network.

U-net++ can be seen as the fusion of four U-net networks of different depths.

The network structure is shown in Figure 2. The left side is downsampled, and each downsampling will be fused with the upper layer, from left to right, and from top to bottom. The blue and green parts in the above figure are the added parts of U-net++ relative to U-net [9, 10]. There are four layers of *L*1–*L*4 with different depth settings on the right side. The black arrow is the same downsampling as U-net. The direction of the blue arrow is the jumper structure. Each horizontal layer is the DenseNet structure, and each prototype unit represents the convolution + activation function [5, 11].

### 3.2. Experimental Operation Based on U-Net++

1. First, after the grape leaves are marked with data, a .json file will appear. The processed .json files are classified into different folders, and the corresponding images and labels are copied to the corresponding folders [11, 12].
2. A data generator is created for model training, Create a data generator for model training, set path of the path reading, and the path is text.train in the above figure. The training size (target_size) is set to 256 *∗* 256 and judged whether the data need data enhancement: valid = ? A zero is used before decimal points—“0.25,” not “.25”—and “cm^3^” is used instead of “cc.”
3. The evaluation metrics of confusion matrix is calculated in the training set, then the confusion matrix is inputted to calculate PA, mPA, and MIOU (average intersection-over-union ratio), and the backbone encoder selects ResNet18 for data processing and feature extraction. The optimizer uses AdamW learning rate denoted as 2*e* – 3 and regularization denoted as 1*e* − 3, and the loss function uses cross entropy to calculate the loss value to train the model. In the final output, the image needs to be resized to restore the original image size, and then the reverse conversion channel and normalization operation are performed. Since the original image is a three-channel color image, the prediction is copied back to the three-channel color image [12].

Next, we use the U-net++ model for image segmentation of grape leaves and compare with traditional OTSU threshold segmentation method (Figure 3).

## 4. Analysis of U-Net++ Experimental Structure Results

The training set first sets the size of each batch of data to 32 (BATCH_SIZE = 32), and the epoch is set to 50. The obtained experimental results use the plot function to obtain a visual training effect diagram. An output folder is created and the segmented images are placed in the output file.

After U-net++ segmentation [13–21], the effect is shown in the figure, and the background is set to black and the pixel value is 0. The model after U-net++ segmentation only retains the part of the grape leaves, without the influence of background noise and other factors.

### 4.1. Model Evaluation

#### 4.1.1. Confusion Matrix

In the field of computer vision, the confusion matrix, also known as the table of possible errors or the error matrix, is a specific matrix used to present the visualization of the algorithm, generally used in supervised learning. Each column represents the predicted value, and each row represents the actual category.

Assuming that there are *n* + 1 categories (including background), the actual category is represented by *Pii* as the *i*th category, and the predicted category is also the *i*th category, consisting of true positive (TP) and true negative (TN). *Pij* indicates that the actual category is the *i*th category, and the predicted category is also the *j*th category, which includes two cases, namely false positive (FP) and false negative (FN) [3, 7]. The confusion matrix is shown in Table 1.

#### 4.1.2. Pixel Accuracy (PA) and Average Pixel Accuracy (mPA)

The ratio of the correct number of pixel classifications to the total number of all pixels is called the pixel accuracy, and the formula is expressed as:

(1) $$\begin{array}{c} PA=\frac{\sum_{i}^{n}Pii}{\sum_{i=0}^{n}Pii\sum_{j=0}^{n}Pij}. \end{array}$$

The confusion matrix calculates the pixel classification accuracy by the ratio of the sum of the diagonal elements to the sum of all elements of the matrix.

(2) $$\begin{array}{c} PA=\frac{\text{TP}+\text{TN}}{\text{TP}+\text{TN}+\text{FP}+\text{FN}}. \end{array}$$

The average accurate pixel rate is to calculate the classification accuracy of each category, and then accumulate the average.

(3) $$\begin{array}{c} \text{MPA}=\frac{1}{n+1}\sum_{i=0}^{n}\frac{Pii}{\sum_{j=0}^{n}Pij}. \end{array}$$

#### 4.1.3. Average Crossover Ratio (MIOU)

The definition of MIOU is to calculate the ratio of the intersection and union of the two sets of the true value and the predicted value, which can be transformed into the sum of Tp (intersection) and TP, FP, and FN.

(4) $$\begin{array}{c} \text{MIOU}=\frac{1}{K+1}\sum_{i=0}^{k}\frac{Pij}{\sum_{j=0}^{k}Pij+\sum_{i=0}^{k}Pij-pii}. \end{array}$$

*Pij* is the number of true values and predicted values of *j*, *K* + 1 is the number of categories, and *Pij* is the real number. *Pij* and *Pji* are false positives and false negatives, respectively.

MIOU is generally calculated based on the class. The IoU value of each class is calculated and then accumulated. After the accumulation, the average is obtained, and the overall evaluation of the model is obtained.

This article uses the plot function to visualize the values of PA, mPA, loss, and MIOU. The significance of the plot function is that the data can be intuitively represented in terms of quantity and trend.

As shown in Figure 4, judging from the fit of the loss function, the U-net++ model has not been overfitted, and the loss value is still at a low level when the epoch reaches 50, with a value below 0.34. Both the PA value and the mPA value are close to 0.99, indicating that the accuracy of the segmented grape leaves is very high, and the proportion of correctly marked pixels in the total pixels is close to perfect [3, 22]. The MIOU value is judged by the evaluation index. The segmentation effect of grape leaves based on U-net++ can well meet the needs of this article for the segmentation of grape leaves in complex environments.

### 4.2. Comparison between Traditional Image Segmentation Methods and U-Net++

Since the result of traditional image segmentation is a binary image, we need to convert the obtained binary image into an RGB color image of the original image [23]. There are two conversion methods. One is to convert the segmented image. One is to restore the segmented image and the orignal imageby the point multiplication operation, and the other is to restore the pseudocolor image. The formula for binarization to restore the pseudocolor image is as follows:

(5) $$\begin{array}{c} R^{\prime }=R\times \text{IBW,}\\ G^{\prime }=G\times \text{IBW,}\\ B^{\prime }=B\times \text{IBW.} \end{array}$$

*R*′ is the red channel of the false color, *G*′ is the green channel of the false color, *B*′ is the blue channel of the false color, and IBW is the binary image of the grape leaves.

Figure 5 is the extract green channel binarized image.

The new *QR* (segmentation algorithm accuracy) and *D* are introduced into the evaluation indicators to evaluate the two indicators of *OR* and *UR*. The larger the value of *QR*, *OR*, *UR*, and *D* is to evaluate the segmentation performance, the better the segmentation effect [24, 25]. The formula of the evaluation index is as follows:

(6) $$\begin{array}{c} QR=\frac{C_{s}}{Os+U_{s+C_{s}}},\\ OR=\frac{C_{s}}{C_{s}+O_{s}},\\ UR=\frac{C_{s}}{U_{s}+C_{s}},\\ D=\sqrt{\frac{UR^{2}+OR^{2}}{2}}. \end{array}$$

Among them, *C*_*s*_ represents the overlap between the segmentation result and the result pixel of the image and the real result pixel, *O*_*s*_ represents the pixel position where the real result in the image is the background, and *U*_*s*_ is the real result of the position of the wheat ear pixel in the image.

In order to make the evaluation of segmentation more objective, this article compares the threshold segmentation and clustering algorithms with the U-net++ algorithm.  Figure 6 shows the comparison of evaluation indictors.

The segmentation of grape leaves in complex background is carried out, the model of U-net++ is adopted, and the model is introduced. The basic structure of the model and the choice of the compiler are introduced, and four kinds of neural network evaluation indicators are introduced and compared with the traditional segmentation methods [26].

## 5. Segmentation of Grape Leaf Lesions Based on Improved OTSU Algorithm

The U-net++ algorithm needs to label a lot of images when processing, and it is difficult to label the disease spots of grape leaves, and it is difficult to accurately label the parts with adhesion [2, 4]. If the U-net++ method is still used, the amount of manual operations is large, and the accuracy of the effect will not be very good. For lesion segmentation, the OTSU [4, 27] method was used for threshold segmentation.

The OTSU threshold segmentation algorithm has obvious shortcomings, and it is too sensitive to image noise. Because the original image of grape leaf lesion segmentation has noise interference from complex environments, we have segmented the grape leaves as a whole when processing the algorithm. The segmentation of the foreground and background is carried out, which shows that the effect of the application is more obvious in images with a large gap between the foreground and background. Therefore, the improvement of the OTSU algorithm is to increase the gap between the foreground and background.

In this article, the segmentation of lesions is based on the U-net++ network for grape leaf segmentation, and after the grape leaves have been segmented, OTSU threshold segmentation [6, 27, 28] is performed on the resultant image [25, 28]. So, the foreground background of the image becomes the diseased spot and the green part of the grape leaves. In this article, the disease classification of grape leaves is also based on the ratio of the area of the two to the total area of grape leaves.

The RGB color system is a color standard in the industry. *R*, *G*, and *B* correspond to three components of red, green, and blue, respectively. An RGB image can be regarded as a stack of three gray images [23, 29].

For an RGB image of grape leaves, the *G* vector of the leaves, that is the green part, is more prominent, and the method of increasing the proportion of the green vector in the image can be used when segmenting grape leaves. First, the color RGB image is processed by ultra-green molecules (2*G*-*B*-*R*) to increase the proportion of green components in the color space. To achieve the ability to enhance the contrast between the *G* component and the *R* and *B* components, the image is then subjected to OTSU threshold segmentation, and the threshold *T* is automatically selected to be compared with the gray value of each pixel [28, 30, 31]. If it is greater than *T*, the target is marked. The rest are used as background. In actual operation, the threshold can also be selected according to experience to achieve the best effect [23, 32, 33].  Figure 7 shows the EXG image of grape leaves.

As can be seen from the comparison of the above figure, the segmentation of the image becomes accurate and reasonable after the EXG ultra-green processing of the image. Similarly, if we use the EXR algorithm to process the lesions of the red vector, the lesions can be segmented. Using the EXR threshold segmentation method to segment the lesions will have an obvious over-segmentation phenomenon, while the EXG algorithm for green vectors will not appear similar to the segmentation of healthy leaves [29, 30]. Therefore, the EXG algorithm is first used to segment healthy grape leaves. After segmentation, MATLAB is used to traverse the pixels of the watermelon and segment the diseased image and healthy leaves by point multiplication, as shown in the figure after segmentation [24, 25].  Figure 8 shows the segmentation process of grape leaf lesions.

From the comparison of Figure 3, it can be seen that it is difficult to completely remove the shadow and noise of the image using the traditional OTSU threshold segmentation method, while the U-net++ method can make the image more accurate and complete.

Therefore, segmenting the green parts or diseased spots of grape leaves is the key to studying grape diseases.

## 6. Grape Leaf Disease Classification

The current grape leaf grading is divided into six grades according to the percentage of disease spots in the leaf area, and the grape leaf disease application program is automatically graded according to the grading table [32]. There are traditional methods used in the study of disease classification of plant leaves. In this article, the traditional disease classification methods are introduced, and the two are compared.

### 6.1. Disease Grading by Traditional Paper Pattern Method

1. Find at least 30 original pictures of grape leaves after segmentation, and print them on hard A4 paper, with three copies of each print;
2. Cut the grape leaves along the edge of the printed leaves and use an electronic balance to measure the paper quality in the leaf area.
3. Trim the diseased area of grape leaves and weigh the remaining paper;
4. Calculate the ratio of the diseased area to the leaf area and obtain the classification result of the leaf disease degree according to the classification standard table.

### 6.2. Disease Grading Using Automatic Grading Method

The grape leaves that have been segmented are converted into a binarized image, because the color of the binarized image has only two colors, black and white, and it is easier to calculate the leaf area [23, 29].

For the calculation of the leaf area, it is calculated according to the pixel points of the target, and the area of the binarized image can be calculated by using the beware function of MATLAB. In the binarized image, the pixel value of the white part of the pixel is 1, the pixel value of the black part is 0, and each pixel point is discrete, so the area formula can be expressed as:

(7) $$\begin{array}{c} \text{Leafareal}=\sum_{i=1}^{M}\sum_{j=1}^{N}f\left(x,y\right), \end{array}$$

where *f*(*x*, *y*) is the binary image of *M* × *N*. Grape disease grading table is as shown in Table 2.

### 6.3. Analysis and Comparison of Test Results

Taking 30 pieces of grape leaf disease collected as the test object, the results after classification were compared with the paper weighing method, and the average error of leaf percentage calculation was about 9.0%. In order to verify the accuracy, the two methods were compared (Table 3) [34, 35].

The percentage of leaf area occupied by the diseased area was tested by *t*-test, and the results showed that there was no significant difference between the two methods (*P* = 0.7117). The accuracy of judging the severity of 30 disease images was 93.33%, and the accuracy of automatic classification of the severity of disease on a single leaf was high.

## 7. Conclusion

This article combines the current common disease segmentation methods of plant leaves and deep learning technology to solve the problem of how to segment all plant leaves, including grape leaves, in complex backgrounds, and from the perspective of segmentation accuracy. Using U-net++ for grape leaf segmentation has excellent results and can completely solve the segmentation problem in complex environments.

When calculating the ratio of the lesion area to the total leaf area, the improvement of the traditional segmentation method was used to deepen the green vector part, and the lesion was successfully segmented. Drawing on the traditional paper pattern method for disease grading, the paper pattern method and the automatic grading method are compared, and the comparison shows that the two conclusions are the same, but the automatic grading method is more flexible and convenient.

## Figures and Tables

**Figure 1:** Grape leaf label.

**Figure 2:** Network structure.

**Figure 3:** Comparison of different segmentation methods. (a) Original picture of grape leaves, (b) after OTSU processing, (c) after U-net++ processing, (d) original picture of grape leaves, (e) after OTSU processing, (f) after U-net++ processing, (g) original picture of grape leaves, (h) after OTSU processing, (i) U-net++, (j) grape leaves, (k) OTSU, and (l) after U-net++ processing.

**Figure 4:** U-net++ network structure evaluation index.

**Figure 5:** Extract green channel binarized image.

**Figure 6:** Comparison of evaluation indictors.

**Figure 7:** EXG image of grape leaves.

**Figure 8:** Segmentation process of grape leaf lesions (a) original picture of grape leaves, (b) partial binarization image of diseased spots on grape leaves, and (c) grape leaf lesions.

**Table 1:** Confusion matrix.

Confusion matrix		Actual value	
		Positive	Negative
Predictive value	Positive	True positive (TP)	False positive (FP)
	Negative	False negative (FN)	True negative (TN)

**Table 2:** Grape disease table.

Severity level	Healthy area of grapes in the total area
0	*s* = 100
1	95% ≤ *s* < 100%
3	90% ≤ *s* < 95%
5	80% ≤ *s* < 90%
7	50% ≤ *s* < 80%
9	*s* < 50%

**Table 3:** Test results.

Paper sample weighing						Automatic grading method	
Num.	Healthy area as a percentage of leaf area					Healthy area as a percentage of leaf area	Level
	1	2	3	Ave.	Level		
01	75.0618	75.7436	75.6156	75.4737	7	75.4197	7
02	87.1972	87.9167	87.4222	87.5120	5	86.8553	5
03	91.2692	91.0336	91.4708	91.2579	3	92.0151	3
04	85.5914	86.0974	86.1686	85.9525	5	87.0481	5
05	84.7540	85.0254	85.1021	84.9595	5	86.8249	5
06	93.8229	93.2244	93.6519	93.5664	3	94.5297	3
07	84.4904	84.5946	84.7279	84.6043	5	84.7958	5
08	86.5663	86.2026	86.3131	86.3607	5	84.6096	5
09	87.9731	87.3498	87.0458	87.4562	5	88.9899	5
10	95.4107	95.3266	95.2586	95.3320	1	95.8372	1
11	88.6523	87.3376	86.7459	87.5786	5	86.7234	5
12	92.3482	91.9691	91.8969	91.8969	3	92.8052	3
13	73.6560	73.9251	73.0720	73.5510	7	76.8400	7
14	81.9866	82.203	81.9470	82.0453	5	84.5947	5
15	94.7682	94.8427	93.8203	94.4771	3	93.6705	3
16	95.5729	95.3866	95.1410	95.3668	1	95.4278	1
17	93.7455	93.4621	93.4322	93.4566	3	92.8014	3
18	88.7826	88.6681	88.8137	88.7548	5	87.1124	5
19	88.0318	88.4044	88.4077	88.2813	5	88.1554	5
20	88.4121	88.2531	88.0640	88.2431	5	89.6066	5
21	87.4235	87.1289	87.1606	87.2377	5	88.9663	5
22	70.8212	70.3008	70.8764	70.6631	7	74.6183	7
23	92.4203	92.5355	92.3186	92.4248	3	92.1274	3
24	87.2165	87.1451	87.0346	87.1321	5	88.2682	5
25	95.0475	95.3197	95.4456	95.2720	1	95.5936	1
26	89.6657	88.7892	88.7813	89.0787	5	89.9492	5
27	95.6244	95.3983	95.2925	95.4384	1	94.8089	1
28	90.1715	90.2095	90.00091	90.1300	3	89.6163	3
29	82.5044	82.4174	82.4824	82.4681	5	83.9878	5
30	89.1660	88.9740	88.8984	89.0128	5	89.6027	5

## Data Availability

The dataset can be accessed upon request.
